# Machine learning-based anomaly detection and prediction in commercial aircraft using autonomous surveillance data

This article has been retracted.

**DOI:** 10.1371/journal.pone.0317914

**Published:** 2025-02-06

**Authors:** Tian Xia, Lanju Zhou, Khalil Ahmad

**Affiliations:** 1 School of Intelligent Manufacturing, Tianjin Electronic Information College, Tianjin, China; 2 School of Instrumentation and Optoelectronic Engineering, Beihang University, Beijing, China; National University of Sciences and Technology, UNITED KINGDOM OF GREAT BRITAIN AND NORTHERN IRELAND

## Abstract

Regarding the transportation of people, commodities, and other items, aeroplanes are an essential need for society. Despite the generally low danger associated with various modes of transportation, some accidents may occur. The creation of a machine learning model employing data from autonomous-reliant surveillance transmissions is essential for the detection and prediction of commercial aircraft accidents. This research included the development of abnormal categorisation models, assessment of data recognition quality, and detection of anomalies. The research methodology consisted of the following steps: formulation of the problem, selection of data and labelling, construction of the model for prediction, installation, and testing. The data tagging technique was based on the requirements set by the Global Aviation Organisation for business jet-engine aircraft, which expert business pilots then validated. The 93% precision demonstrated an excellent match for the most effective prediction model, linear dipole testing. Furthermore, the "good fit" of the model was verified by its achieved area-under-the-curve ratios of 0.97 for abnormal identification and 0.96 for daily detection.

## 1. Introduction

Flights are an essential part of modern society forgetting about. More people are taking to the skies, which proves this. The rising demand for commercial aircraft and associated services was the subject of an investigation, as demonstrated by [1]. Many unanticipated limitations pertaining to wellness, the internet, the natural world, and security have arisen as a consequence of the dramatic rise in transportation demands and the aspirations of users to shorten journey times. The security of the aviation industry is critical. The worst disaster in Boeing’s history occurred in 2018 when two passenger Boeing 737 MAX 8 aircraft collided, shocking the aviation sector [2]. As a result, accident evaluation has taken the front stage. When looking into plane crashes, investigators first looked for the black box that contains the flight records (FDRs) and the pilot’s recording devices (CVRs) [3]. In order to protect their homelands and valuable assets, European countries ramped up their technological abilities during World War II (1939–1945). Len Harrison and Vic Husband, two British scientists, designed a crash and fireproof flight record for the UK’s Ministry of Aviation Production. According to the Centre and Copyright (2020), this innovation has now set the standard for this sector. The use of both analogue and digital information types in black boxes has evolved to assist with aircraft crash investigations [4]. An aircraft recording device (CVR) is a piece of aircraft equipment that records and stores all of the audio from the cockpit, including voice conversations, radio broadcasts, and background noise. This device is designed to endure the force of a collision while protecting the information that has been collected. A number of flight operating parameters, including the speed of the air height, headings, vertical speed, sensor readings, flight-control actions, and engine efficiency, are continuously recorded by an aircraft’s crash-proof Flights Information Record (FDR) [5].

In examinations into aviation accidents, the black box—which is renowned for its ample storage of information capacity—has become an indispensable tool [6]. Both primary and secondary sources were the two main types of data [7]. Even though it has its limits, the primary data kept in the black box is still used as the primary reference. Data retrieval after black box destruction requires a specific interface. Depending on the circumstances, this can take some time to happen [8]. The United military government began developing the next generation of air transport system (NextGen) in 2005 to address this issue. The goal of the programme is to use digital signal relay technology from aeroplanes to make air travel more efficient, safer, and more predictable (FAA, 2020). Automatic dependant surveillance-broadcast (ADS-B) is a new technology that the CIA introduced as a substitute for radar. With ADS-B, aircraft may use a global navigator to find themselves without human intervention. It also facilitates interaction among planes and planes on Earth by relaying vital data like speed, guidance, height, and others via electronic links [9].

Additional information has been made available by the gathering of flight data by ADS-B [10]. The development of a machine-learning model for the detection and prediction of commercial aeroplanes using data from ADS-B technologies is crucial for the reduction of crashes involving aircraft. The primary goal of this research is to find any anomalies in the departure and ascent conduct of business aircraft that could lead to the prevention of plane crashes. When looking into aircraft mishaps, ADS-B data is utilised with black box data. In order to forecast future flying data, machine training (ML) is used to examine previous flight information from commercial aeroplanes. [11, 12] are only a few of the studies that have looked at the trends of flight behaviour utilising data recorded by the systems on board rather than black boxes. In this research, we built a model using machine learning that incorporates all three parts of the survey: identifying ADS-B quality of data, detecting anomalies, and categorising irregularities.

This study significantly contributes to the literature by advancing the application of machine learning for anomaly detection and accident prediction in commercial aviation. By leveraging data from autonomous surveillance systems like ADS-B, the research bridges a critical gap in the aviation industry, focusing on real-time monitoring and predictive modeling. The development of abnormal categorization models tailored to business jet-engine aircraft enhances the understanding of flight irregularities and their potential precursors, thus contributing to aviation safety. The methodology, which integrates data selection, tagging based on ICAO standards, and expert validation, ensures a robust framework for model development and evaluation. Achieving a precision rate of 93% and high area-under-the-curve values (0.97 for abnormal identification and 0.96 for daily detection) showcases the model’s efficacy, setting a benchmark for future studies. This work not only underscores the importance of using advanced statistical and machine learning techniques in aviation safety but also provides a scalable framework for proactive anomaly detection and mitigation strategies. By integrating practical insights with theoretical advancements, the study contributes to the evolving discourse on AI-driven safety measures, offering a novel perspective and potential applications for flight safety and operational efficiency in the aviation industry.

There are several sections to this text. Included in the beginning are the research’s background, objectives, and current standing. The next step was a review of the relevant literature, which included the development of the research’s underlying assumptions. The following section is the Material and Techniques, which consists of the sources of information and the procedures utilised to achieve the goals of the research. The paper is divided into three primary parts: The research’s three sections are as follows: leads to and debate, which gives the research’s results and discusses them; conceptual and managerial consequences, which looks at how the findings could affect theory and leadership in travel safety; and the end, which concludes the research.

## 2. Literature review

There are a lot of uses for machine learning (AI), including improving flight paths, anticipating when engines will fail, and giving customers virtual assistance. Improvements in the efficiency of operations, security precautions, and customer service quality have been caused by the deployment of AI in commercial airlines [13]. Aircraft may save time and fuel by using AI to analyse weather and flying data and determine the most effective paths [14]. The application of machine learning (AI) in engine problem prediction has allowed carriers to perform repairs and decrease flight delays preemptively [15]. In addition, digital assistants powered by AI are soon to be available to handle customer service queries, help with ticket purchases, and offer flight information (TAV Technologies, 2023). According to [16], it is clear that artificial intelligence uses for business aircraft are now and will continue to progress. Data is used in the specific field of machine learning, or ML, to teach machines to detect trends, make forecasts, and act autonomously [17]. In order to examine data and find patterns, artificial intelligence makes use of multiple algorithms and statistical approaches. Researchers have turned to machine intelligence (ML) as a means to analyse massive amounts of past information for trends or insight because of this capability and technological improvements. They may be able to use these findings to solve complex problems (Sarker, 2021b). Research on the use of artificial learning to foresee various flight features, including cancellations and interruptions, is growing. According to [18], ML models are used to predict probable cancellations and delays in flights by analysing past data, such as weather trends, terminal illnesses and aircraft movements. The ability to proactively inform customers, reschedule flights, and reallocate personnel is a boon to carriers.

Another research [19] utilised ML to predict how much fuel aircraft will consume. In order to improve the precision of fuel use forecasts, the algorithm considers factors including flight paths, weather, and aeroplane types. Research by [20] suggests that airlines may save costs and reduce emissions of dioxide into the atmosphere by employing this strategy. The prediction of engine failure in aeroplanes has also made use of artificial intelligence. The programme analyses data gathered from aeroplane engines’ sensors to detect early warning signs of damage and predict the likelihood of failure. Because of this, airlines may prevent accidents by performing routine safety steps. That is according to [3]. Thanks to the increasing usage of ADS-B data in aviation in the digital era, researchers have been motivated to investigate flights for commercial use. Scientists have utilised ADS-B data for a variety of business flight-related investigations, including air traffic management. Increased security during flight and the detection of potential issues are both made possible by the technology’s real-time surveillance of aircraft movement. It may also identify areas with a high number of people and monitor trends in air traffic.

As a result, aviation regulators are able to control air better. Also, the journey was made more efficient with the use of ADS-B data. Airline companies may save money on time and fuel by analysing flight paths to find the most economical ones. Using ADS-B data optimises aircraft shifts, increases flight reliability, and enhances the accuracy of plane time of arrival projections. A recent innovation is the use of ADS-B information in crash investigations. In order to better understand what happened and how to prevent future mishaps, researchers may use ADS-B information to simulate flight conditions. Before the plane’s black box can be retrieved, the investigation into the crash begins with using ADS-B data for this simulation [21]. Additionally, airlines may use this data to evaluate pilot and aeroplane efficiency, which can help them improve safety measures and instruction [22]. The purpose of this software is to analyse flight patterns. Aircraft rises and descends, among other flight trends, are being evaluated using ADS-B data. In addition to analysing flight equipment faults, this will help airlines improve fuel economy and limit emissions. There are many benefits and promising future possibilities for airlines to use ADS-B data for business aircraft-flight analytics. Airline security, effectiveness, and environmental responsibility are all improved with the adoption of ADS-B technology. Table 1 provides a synopsis of the studies done on ADS-B data processing and analysis. There has been a recent uptick in studies examining the use of ML in business aviation, with a focus on ADS-B data. In the following years, the aviation sector is expected to reap multiple advantages from this research.

**Table 1:** A small number of research that rely on ADS-B data.

Citation	Title	Problem	Method	Result	Limitations
[23]	Research of ADS-B data evaluation	Evaluating the performance of ADS-B for coordinating data from several sensors.	Estimation of future data using higher update rates from lower ones.	ADS-B outperforms radar in terms of performance.	Limited to specific scenarios with high update rates; broader validation needed.
[24]	Analysis of anomalies in ADS-B and its GPS data	Issues with GPS data in ADS-B due to primary and secondary radar discrepancies.	Statistical analysis of GPS and radar comparisons.	Existing ADS-B system has several flaws that must be addressed before reliable implementation.	Did not propose concrete solutions for GPS-related ADS-B discrepancies.
[25]	Investigation of the effects of ADS-B and radar on DAA systems	Determining how often and for how long radar and ADS-B systems experience communication failures.	Statistical analysis of the frequency and length of communication outages in discrete intervals.	Neither radar nor ADS-B data exhibited any loss of transmission.	Limited scope; does not explore performance under noisy or degraded conditions.
[26]	Discrepancies in UAT ADS-B data and their impact on dropouts	Understanding how UAT ADS-B data irregularities affect ATC operations.	Statistical methods and Friedman tests applied to data.	Found 32.49% data inconsistency due to dropouts and other irregularities like interruptions.	Does not address potential mitigation strategies for dropouts.
[27]	Checking the availability of ADS-B data sources depending on precision	Assessing the quality and accuracy of ADS-B signals for ground and flight crews.	Simulation validation of airport data and analysis of navigational data sources.	Confirmed that ADS-B airport navigation sources meet required accuracy standards.	Results based on simulations rather than real-world validation.
[28]	Exploring ADS-B data from regular helicopter tours for new insights	Identifying patterns in helicopter flight data using ADS-B.	Statistical analysis and clustering methods applied to flight trajectory parameters.	Subject-matter experts used results to identify trends for anomaly detection in flight records.	Focused solely on helicopter data; lacks generalization to fixed-wing aircraft.
[29]	Identification of activities at aviation-related airports using ADS-B	Differentiating flight operations and activities at smaller airports using ADS-B data.	Classification of aircraft data collected from smaller airports using AWS as a data platform.	Successfully labeled flights with their operating types after completing classification procedures.	Limited to smaller airports in the US; lacks global applicability.
[30]	Safeguarding pilots and flight data in an ADS-B environment	Enhancing ADS-B systems to strengthen pilot safety and flight data integrity.	Advocating digitization programs and real-time data transmission from takeoff to landing.	Stressed the need for enhancing ADS-B and other aviation technologies urgently.	Focused on high-level recommendations without providing technical implementation details.
[31]	Energy anomaly identification using isolation forest on ADS-B data	Improving safety in civil aviation by detecting anomalies in energy data using ADS-B flight data.	Application of isolation forest algorithm (iForest) to detect anomalies iteratively.	Successfully identified energy anomalies in ADS-B trajectory data.	Does not consider false positives or robustness of iForest under varying conditions.

## 3. Materials and methods

### 3.1. Data sources

Preparing data from studies is an essential first step in conducting scientific studies and building models for forecasting. Before building prediction models utilising artificial intelligence methods, scientists must carefully gather and prepare data to guarantee the precision and validity of the outcomes. There are obstacles to this procedure. In this section, the difficulties and basic methods of data preparation for the research are discussed. The initial step was to collect flight records found in the ADS-B database. The serious events that happened during the years 2018 and 2019 had an impact on the choice of B737 Maximum 8 data. According to [32], this specific type of aircraft was subsequently banned from March 2019 until the end of 2020. All of the information that has been provided above comes from aircraft databases like, which is a Flightradar24. The primary goal of this research was to highlight the need to carefully consider a wide range of factors when selecting data sources in order to ensure high-quality data. [33] all stress the need to use ADS-B data that follows accepted guidelines in order to get reliable results. Business aeroplane ADS-B data is comprehensively available in the OpenSky Networks repository. The B737 MAX 8 system is a good illustration of this kind of system. Data from 167,844 B737 MAX 8 travel, including departure and rising, make up the data set. All three types of data—training, testing, and validation—are at your disposal. This dataset is in CSV format and has a size of 6 GB. [34] have both published the data. Prior to cleaning and information labels, the ADS-B data is combined into a single database.

### 3.2. Preparing files and tagging data

The original dataset consisted of eight factors, including time, callsign, latitude, longitude, barometric altitude (baroaltitude), speed, heading (going), and period. During the data preprocessing stage, a feature-selection procedure was applied to refine the dataset and retain only the most relevant variables for analysis. As a result, five key factors—timestep, baroaltitude, speed, heading, and period—were selected, while others such as callsign, latitude, and longitude were excluded due to their limited relevance to the research objectives. This refinement ensured that the analysis focused on the parameters most critical for detecting anomalies and predicting aircraft behavior effectively. The data preprocessing and labeling methods in this study were carefully designed to ensure the reliability and validity of the machine learning model for anomaly detection. Data preprocessing involved cleaning the raw ADS-B data to remove noise, inconsistencies, and irrelevant variables, followed by feature selection to retain only the most informative parameters, such as barometric altitude, speed, and heading. These parameters were chosen based on their significance in capturing anomalies during the takeoff and ascent phases of commercial aircraft. The labeling process relied on predefined thresholds derived from industry standards and expert inputs. For example, changes in barometric altitude exceeding 100 feet within a 10-second interval were labeled as abnormal, as such variations are indicative of potential operational issues. This threshold was further validated by commercial airline pilots with Airline Transport Pilot Licenses (ATPLs), ensuring domain expertise was incorporated into the labeling process. The dataset was then split into training, testing, and unseen validation sets to assess the model’s performance comprehensively.

In relation to existing literature, this study addresses several gaps. While prior research has focused on ADS-B data for monitoring flight operations and identifying trends, few studies have implemented machine learning models tailored for anomaly detection during specific flight phases. The integration of real-time ADS-B data with machine learning techniques, such as Quadratic Discriminant Analysis (QDA), fills this gap by providing a framework that is both proactive and precise. Compared to earlier studies, this work stands out by demonstrating high accuracy (93%) and robust AUC values (0.97 for anomaly detection), underscoring its practical applicability in aviation safety. Furthermore, the study contributes to the literature by emphasizing data preprocessing and labeling techniques that ensure the model’s generalizability and reliability. These findings not only validate the use of ADS-B data for anomaly detection but also pave the way for future research to extend these methods to other flight phases and parameters, thus addressing the broader challenge of enhancing aviation safety through data-driven approaches.

Signs of distress are unnecessary since the data records have been organised according to the trip. In addition, the dataset did not include the GPS variables (latitude and longitude) since they were considered unimportant in the absence of flight-trajectory information. Attributes from each of the five established factors were selected to form the desired factor. Time and baroaltitude are strongly positively associated, according to Pearson’s correlation value of 0.894417. To elaborate, as indicated in Table 2, the aeroplane’s elevation or baroaltitude appears to increase with time. The research’s variable of dependence, baroaltitude, was so selected.

**Table 2:** Specific details regarding the ADS-B data file format used by commercial aircraft.

*Time step*	*Time*	*Baroaltitude (feet)*	*Velocity (knots)*	*Heading (degree)*
0	1504225932	100.92	2	28.82
10	1504225942	283.52	79.32	28.23
20	1504225962	435.52	82.02	2.12
30	1504225993	511.102	94.702	359.22
40	1504226033	647.702	101.91	358.74
50	1504226083	815.342	111.61	319.03
60	1504226143	1106.992	112.21	287.43
70	1504226213	1372.172	115.51	253.03
80	1504226293	1615.502	116.91	219.23
90	1504226383	1875.612	115.01	187.13
180	1504226563	11704.32	250.52	88.83

Direction, speed, baroaltitude, timestep, and length are the five parameters that comprise the voyage information format shown in Table 2. Because it affects later steps, understanding and investigating the data distributions is also critical. An essential part of data analysis is the exploratory data analysis, or EDA, phase. Finding connections, trends, and outliers required an initial data analysis. Developing ideas and guiding additional studies are common uses of the EDA. EDA uses many traditional approaches: Descriptive statistics are used to provide a clear and concise summary of the data. The median, mean, and mode are three measures of centring that are used to characterise the usual values of a parameter. We use dispersal measures like volatility and median deviation to show how dispersed the data is. While time data follows an average dispersion with 0% skew, baroaltitude data shows aberrant shipping, according to the results. The next step included selecting 3,000 flight information points randomly. Then, we calculated the intervals among all of the observational data points. According to many sources [35], the difference in height was determined to be more than 100 feet within a 10-next time frame. When taking off and navigating, business aeroplanes must keep their movements stable, which is why stability is so important. Descending over 100 metres in just over a minute causes air-pressure disturbances and irritation in the cabin. Any altitude shifts more than 100 feet throughout a 10-next timeframe will be considered abnormal in the cockpit data. Two thousand cases were marked as abnormal, and one thousand were categorised as typical out of three thousand ADS-B flight records that made up the collection. Pilots from commercial airlines in the country with airline transport-pilot licences (ATPLs) and at least 1500 flight hours were then asked to verify these details. After over two months of testing, we were able to validate that each of the three thousand points of data had been properly tagged and were suitable for use. Once the 164,844 flight points of data were tagged, the next phase was to classify and differentiate between abnormal and standard information. The two aeroplane data given to the expert include baroaltitude as well as time data points ranging from the launch phase through the ascending stage (Fig 1). The difference between abnormal and typical information is shown graphically in the figure.

**Fig 1:** Shows the representation of both typical and out-of-the-ordinary data.

There were 167,844 data points (flights) analysed using the data labelling approach; 84,074 were classified as usual, whereas 83,770 were classified as problematic. Following normalcy and atypicalcy annotations, the data was divided into train and testing sets. In order to build a machine learning model, the classification is vital. The dataset’s unique characteristics and the chosen artificial intelligence models dictate the data classification strategy. There are 167,844 flights in the collection; 84,074 are considered acceptable data, and 83,770 are considered questionable. The data was also partitioned using random sampling, with 30% being test flight information and 70% being training information. With no unknown information included, the result produced 117,490 data points to use as training and 50,354 information points for testing. The Flightradar24 site was used to get previously unseen data. Undetected data was created using the same process as the database, incorporating test and training data (Passarella & Nurmaini, 2022). For a detailed rundown of each data partition, see Table 3.

**Table 3:** The data set used to build the prediction model and its components.

Parameter	Normal	Abnormal	Subtotal
*Training*	58,781	58,718	117,491
*Testing*	25,291	25,012	50,351
*Unseen*	1001	1001	2001
*Subtotal*	85,014	84,771	–
*Total dataset*	–	–	169,817

The unbalanced ratio was computed to characterise the degree of instability in a dataset. According to [36], the incorrect ratio was determined using a preset method, shown in Eq (1). The data equilibrium among the training and testing groups was determined using Eq (1). As seen in Table 4 the dataset exhibited balanced features according to the computations. One may tell if the model they have picked is correct when the imbalanced ratio comes near 1.

**Table 4:** Table displaying the outcomes of the unbalanced ratio computation on the dataset.

Dataset	Normal	Abnormal	The imbalance ratio	Remarks
Training	58,782	58,708	1.009	Balanced dataset
Testing	25,292	25,062	1.009	Balanced dataset


$$Theimbalanceratio=\frac{N_{maj}}{N_{min}}$$ (1)

The size of the minority class is denoted by Nmin and the size of the majority sample is Nmaj in expression (*N*_*maj*_).

### 3.3. Method

The study presents a machine learning-based model for anomaly detection and prediction in commercial aircraft, demonstrating clear advantages over other models in the field. Among its key advantages is the use of Quadratic Discriminant Analysis (QDA), which outperformed 25 alternative machine learning models in terms of accuracy, precision, and computational efficiency. The QDA model achieved a high accuracy rate of 93% with area-under-the-curve (AUC) values of 0.97 for anomaly detection and 0.96 for normal operations, making it a "good fit" for the data. Its ability to deliver precise predictions with a lower computational time compared to complex algorithms such as Random Forest or Gradient Boosting enhances its practical applicability in real-time scenarios. Furthermore, the integration of ADS-B data—an innovative approach compared to traditional reliance on black box data—enables real-time anomaly detection, offering a proactive solution to enhancing aviation safety.

However, the model is not without limitations. One key limitation lies in its dependency on high-quality, labeled data for training, which required extensive expert validation and preprocessing. This process can be resource-intensive and time-consuming, potentially limiting the scalability of the approach for different types of aircraft or operational scenarios. Additionally, while the model performs exceptionally well with ADS-B data, it is primarily validated for a single parameter—barometric altitude—which may not fully capture the complexities of flight anomalies influenced by factors like speed, direction, and weather conditions. As such, the model’s generalizability to other flight phases or diverse datasets might require further enhancements and validation. Despite these limitations, the study provides a robust framework for anomaly detection, paving the way for future research to address these challenges and expand its applicability.

Typically, the process of creating abnormality-prediction systems for business aeroplanes using machine learning involves many steps. During the initial phase, the data set acquired via OpenSky was scrutinized for anomalies and then categorized before receiving validation from a qualified professional (a professional pilot). The authenticated data is then transformed into the data set for utilization. In addition, the whole set underwent processing, and the results were divided into testing and training sets, which were then used to create classification algorithms. For the above model construction, a total of 25 methods were used. Subsequently, the most optimal models were chosen by evaluating the matrix of confusion, reporting categorization, and cross-validation as For the subsequent phase, flight records that had been omitted from the initial data were used. The procedures used were identical to those used in the initial data set, and the second data was likewise identified and categorized as shown in Fig 2. These data sets were also classified as unknown. The top-performing model achieved during the first phase was assessed using undisclosed data to measure its efficacy. The remaining stage yielded a predictive approach for identifying abnormalities during the descent and ascent periods on business flights. Fig 3 depicts the creation of the method.

**Fig 2:** Propose machine learning model.

**Fig 3:** Shows a machine learning workflow.

## 4. Results and discussion

Utilising the technique above, this part details the most effective model testing, the most excellent choice of model from the 25 models used for training, and the best model validation with unknown information.

### 4.1. Evaluation of the model trained

Education models are essential tools for optimizing student accomplishment while creating and executing a training program. In order to construct prediction algorithms, it is crucial to rely on data-driven training. Data preprocessing, model choice and evaluation, and hyperparameter tuning are three factors that impact the efficacy of AI models. The selected approach must be employed when developing an artificial intelligence model. To facilitate testing and training, the approach partitions the data into a lot of sets. Subsequently, it is necessary to implement the model on the training dataset. The primary factors to consider when picking a training framework are learning objectives, data characteristics, and the strategy for generating a machine model [37]. The models for prediction were derived after an examination of 25 distinct models. The findings of this investigation are shown in Table 5. The evaluative criteria were time to execution, F1 score, ROC (receiver operating characteristic) area beneath the curve (AUC), balanced precision, and precision. The data demonstrated that the model’s quadrant discriminant evaluation (QDA) model had the highest correctness rate of 0.93 and precision rate of 0.93 among all the prediction models. The model required 2.46 seconds to finalize its predictions.

**Table 5:** Evaluation of the created prediction models.

Number	Model	Accuracy	Balanced accuracy
1	QuadraticDiscriminantAnalysis	0.93	0.93
2	NuSVC	0.7	0.7
3	LGBMClassifier	0.58	0.57
4	XGBClassifier	0.57	0.57
5	RandomForestClassifier	0.56	0.56
6	ExtraTreesClassifier	0.55	0.55
7	BaggingClassifier	0.54	0.54
8	LinearDiscriminantAnalysis	0.54	0.54
9	RidgeClassifierCV	0.53	0.53
10	RidgeClassifier	0.53	0.53
11	CalibratedClassifierCV	0.53	0.53
12	DecisionTreeClassifier	0.53	0.53
13	LogisticRegression	0.51	0.51
14	SVC	0.51	0.51
15	GaussianNB	0.51	0.51
16	NearestCentroid	0.51	0.51
17	AdaBoostClassifier	0.51	0.51
18	SGDClassifier	0.51	0.51
19	BernoulliNB	0.52	0.52
20	ExtraTreeClassifier	0.52	0.52
21	KNeighborsClassifier	0.52	0.52
22	DummyClassifier	0.51	0.51
23	LinearSVC	0.51	0.51
24	PassiveAggressiveClassifier	0.41	0.41
25	Perceptron	0.41	0.41

The model with the most fantastic accuracy and fastest calculation time was chosen. Fig 4 shows the strong performance of the QDA and NuSVC models. Quantum Dot Analysis (QDA) proved to be the fastest and most accurate method. The study presents a comparison of 25 machine learning algorithms in terms of precision, delay, and ROC-AUC, as illustrated in Fig 4. All the algorithms shown in the figure were implemented to ensure a comprehensive evaluation of their performance on the anomaly detection task using ADS-B data. These algorithms include popular models such as Quadratic Discriminant Analysis (QDA), Random Forest (RF), XGBoost (XGB), Extra Trees (ET), Logistic Regression, Support Vector Classifier (SVC), K-Nearest Neighbors (KNN), Decision Tree (DT), AdaBoost, Gaussian Naive Bayes, and Isolation Forest, among others. Each algorithm was trained and tested under the same conditions, using the same dataset split to ensure a fair comparison. Performance metrics such as precision, delay (time taken for predictions), and ROC-AUC were calculated for each algorithm to highlight their strengths and weaknesses. Hyperparameters for each algorithm were either tuned or kept at standard default values where appropriate. Computational efficiency and resource requirements were also considered, particularly to evaluate the suitability of each algorithm for real-time anomaly detection in aviation. Among these, QDA emerged as the best-performing model with the highest precision and ROC-AUC values, coupled with relatively low delay, making it the most suitable for the task. The comparative analysis ensures that the selection of QDA was data-driven and methodologically robust, while also providing insights into how other models performed under similar conditions. This comprehensive approach not only validates the choice of QDA as the best model but also underscores the study’s methodological rigor in exploring a wide range of machine learning techniques for anomaly detection.

**Fig 4:** Comparison of the 25 ML algorithms in terms of precision, delay, and ROC-AUC.

Assuming a customarily distributed distribution for each class is critical to QDA’s generating model. Class-specific prior data represent a small percentage of a class’s observations. According to [38], the subclass-specific mean vector is responsible for averaging the class input variables. By use of a confusion matrix, the results of the QDA predictions were investigated. One way to evaluate ML classification is via an ambiguous matrix. The matrix of confusion that was developed for the QDA system is shown in Table 6. The system gave the correct label, as usual, to 56,787 planes’ data; those are the TPs. The system accurately identified 52,623 flights as anomalous, such as the TNs.

**Table 6:** Matrices that cause confusion when training the QDA.

*Parameter*		*Predicted label*	
		*Normal*	*Abnormal*
*True Label*	*Normal*	56,781	1991
	*Abnormal*	6081	52,621

Table 7 displays the disarray in the matrix categorization result. The accuracy level was 0.90 using 58,782 typical points of data. The accuracy of the algorithm’s optimistic forecasts is shown by its accuracy, which is an ML success measure. When data is mistakenly labelled as being expected by the device, this is known as a false positive (FP). As seen in Eq (2), *accuracy* is defined as the ratio of true positives (TPs) to the sum of every optimistic forecast (TP + FP).


$$Precision=\frac{TP}{TP+FP}$$ (2)

**Table 7:** Detailed report on the training classification of the QDA prediction model.

Parameter		Precision	False discovery rate	Recall	F1-score	Specificity	#Data
Normal	0	0.9	0.034	0.97	0.93	0.9	58782
Abnormal	1	0.96	0.103	0.9	0.93	0.97	58708
Accuracy		–	–	–	0.93	–	117490
Macro avg.		0.91	0.0681	0.91	0.91	0.91	117494
Weighted Avg.		0.91	0.0681	0.91	0.91	0.91	117494

Eq (3) may be used to get the classification (false detection) rate if the accuracy value has been determined.


$$Falsediscoveryrate=\frac{FP}{FP+TP}$$ (3)

There was a 3.39 per cent rate of incorrect predictions for the standard label and a 10.3 per cent rate for the unusual label. To get the initial model’s particularity, also known as the real-negative rate, use the following formula: specificity = conditional probability of all test adverse outcomes divided by the number of genuine negatives (TNs) (4).


$$Specificity=\frac{TN}{TN+FP}$$ (4)

### 4.2. Analysis of model testing

Model testing was used to assess the most accurate model chosen from the training data. One step of this approach was making predictions about the labeled test data. Table 3 shows the test data that was used to train the QDA model. It included 25,292 normal data points and 25,062 outlier data points. Using the ambiguity matrix in Table 8, the findings showed a 93% accuracy rate in the testing.

**Table 8:** Equation of confusion for the QDA model with test data.

*Parameter*		*Predicted Label*	
		*Normal*	*Abnormal*
*True Label*	*Normal*	24,464	823
	*Abnormal*	2507	21,565

Table 9 displays the confusion matrix as a report that classifies test results. The model-testing procedure used information from 50,344 aircraft as the standard dataset.

**Table 9:** Prediction model construction and testing classification report for QDA.

Parameter		Precision	False discovery rate	Recall	F1-score	Specificity	#Data
Normal	0	0.91	0,032	0.97	0.94	0.9	25,292
Abnormal	1	0.96	0,092	0.9	0.93	0.97	25,062
Accuracy		–	–	–	0.93	–	50,354	
Macro avg.		0.94	0.062	0.93	0.93	0.93	50,354
Weighted avg.		0.94	0.062	0.93	0.93	0.93	50,354

### 4.3. Applying the cross-validation method to the testing process

Due to the fact that even the optimal model could struggle with novel data inputs, evaluating the generated model’s durability is essential. Verifying that the developed model exhibits minimal bias and variation is necessary. What this implies is that the algorithm is able to detect trends in the data with little distortion. Verification is a method of assessing the reliability of numbers that describe the data by quantifying the believed relationships between factors. Assessing an algorithm’s residual error after training is called residue assessment [39]. Learning error, defined as the percentage difference between predicted and actual results, is computed during this process. Nevertheless, this evaluation considers the model’s effect on its training data; it is conceivable that it may not adequately or excessively match the data. The problem with this kind of evaluation is that it needs to find out how well a student can apply what they have learned to other previously undiscovered data. Hence, researchers from all over the world have proposed using the technique known as cross-validation. There are four different methods for cross-validation: holdout, a K-fold, stratification K-fold, and leave-p-out.

Strategic cross-validation with K-folds was used in the research since it is a very reliable and stable approach for analyzing outcomes. Some of the encoding variables were ten for the K-value, two for the number of repeats in cross-validating, and one for controlling the production of random states for each recurrence, which is known as randomised_state. The testing strategy comprised repeatedly running the divided k-fold procedure with different randomizations in every iteration. Py was used to implement the transmitted cross-validation K-fold method. Numpy and learning were the sources of code that were utilized. The results of the multilayer cross-validation k-fold technique are shown in Table 10. The relationship results (K-Fold) showed that the average F1 score was 0.93, and the average run-repeat accuracy rating for the precision F1-score measures was 0.94. The QDA models have attained an adequate level of accuracy, as shown in Table 10, as the average outcomes of the multilayered K-fold cross-validation coincide with the results of the training and verified model. Transmitter Operating Characteristics (ROC) plots were generated to confirm this.

**Table 10:** Every run (n-repeats) and fold (n_splits) cross-validation score as a whole.

Number of Folds	Accuracy			F1-Score		
	Run 1	Run 2	Run 3	Run 1	Run 2	Run 3
*Fold* 1	0.93	0.93	0.94	0.93	0.93	0.93
*Fold* 2	0.94	0.94	0.94	0.93	0.93	0.93
*Fold* 3	0.94	0.94	0.94	0.93	0.93	0.93
*Fold* 4	0.94	0.93	0.93	0.93	0.93	0.93
*Fold* 5	0.94	0.94	0.94	0.93	0.93	0.93
*Fold* 6	0.94	0.94	0.94	0.93	0.93	0.93
*Fold* 7	0.94	0.94	0.94	0.93	0.93	0.93
*Fold* 8	0.94	0.94	0.94	0.93	0.93	0.93
*Fold* 9	0.94	0.94	0.94	0.93	0.93	0.93
*Fold* 10	0.93	0.93	0.94	0.93	0.93	0.93
*Avg*	0.94	0.93				

### 4.4. A receiver operating characteristic (ROC) plot evaluation of the actual positive and false favorable rates

ROC charts are often used when testing the efficacy of a system of classification. ROC curves are helpful in finding the best categorization cutoff since they graphically show the connection between an algorithm’s accurate positive outcomes and favourable error rates. Examining ROC charts, contrasting the true positive with false favourable rates, and explaining their relevance in evaluating models of classification are the main topics of this chapter (Streiner & Cairney, 2007). The results of a model for classification may be seen visually in ROC graphs. They plot the two-dimensional rates of both true and false positives on a graph, where the y-axis shows the actual rate and the x-axis shows the rate of false positives. The ability of the model to differentiate among both positive and negative categories is evaluated in these graphs. An utterly accurate model would have an AUC of 1, whereas a model which is only speculating would have an AUC of 0.5. According to [40], the actual rate of positive outcomes measures how many positive events a model accurately categorized as positive.

To get the result, add up all the good and bad results and then divide that total by the amount of real positives [41]. Cutoff value, number of samples, or positive category prevalence are determinants of the actual positive rate. According to [10], the rate of true positives is an essential metric for models of classification. A higher rate of true positives was required to identify irregularities in this research. Prediction errors are the consequence of a low proportion of right optimistic forecasts and a significant number of erroneous pessimistic forecasts. The percentage of adverse occurrences that the algorithm incorrectly labels as being positive is called the rate of false positives. A simple division of the sum of false positives and genuine negatives by the total number of false negatives is all that is needed for the computation. The predominance of the positive lesson, the sample size, and the threshold value are three factors that impact the percentage of false positives. A critical metric for assessing classification algorithms is the false positive rate, which quantifies how well they detect negative scenarios. Preventing the erroneous identification of genuine transactions as false positives or, conversely, actual transactions as false negatives is a crucial part of detecting fraud. However, costs may increase and unwarranted tests might be justified if there is a high rate of incorrect positives, which could lead to a large number of wrong positive findings. By examining the intersections of the actual positive and false negative rates on the ROC plots, we were able to evaluate the nature of the connection between the two. The optimal threshold is shown by the point where the rates of true positives and false positives meet on the ROC curve. The optimal balance between the rates of true positives and false positives is achieved at this level.

A vertical line, standing for the idea of random speculating, separates the genuine negative rate from the rate of false positives. In order to achieve an appropriate equilibrium between specificity and sensitivity, it is essential to distinguish between the rate of true positives and the rate of false positives. Since it means the model correctly identified a more significant percentage of positive events, a higher actual positive rate suggests the superior performance of the model. When the real affirmative rate is low, it means that the test is exact; in other words, it detects most negative situations correctly. A trade-off is made between both, however, since improving one could have a negative impact on the other. ROC charts help to visualize the trade-off between sensitivity and specificity to find the optimal limit. To compare models for classification, ROC plots look at areas under the curve (AUC) and the difference in true and false favourable rates. For instance, if the area under the curve (AUC) for both models is equal, but one of them has a lower rate of false positives and a higher real-positive rate, it means that the algorithm is better at identifying optimistic scenarios with a lower rate of false positives. Fig 4 displays the findings of the Squared Area Over the Curve (AUC) and Transmitter Operational Characteristics (ROC) plot for the Python-developed Quad Discrimination Analysis (QDA) model. With a capability of 0.97, the model can identify abnormalities.

This system has a normality-detection rate of 0.96. Table 11 shows that the categorical analysis produced reliability values of 0.94 throughout the test and instruction, indicating a good match between the algorithm and the data. Additional validation was sought by generating Transmitter Operational Characteristics (ROC) curves in Fig 5.

**Fig 5:** Area under the curve (AUC) and ROC curves for average, out-of-the-ordinary, and random values.

**Table 11:** A review of the model’s effectiveness.

ML Model Quality	Conditions	Description
Good Fit	• *low bias* • *low variance*	*Accurate and precise predictions*
Overfitting	• *low bias* • *high variance*	Totally different forecasts based on the same data
Underfitting	• *high bias* • *low variance*	Identical data used to generate inaccurate predictions (the algorithm "misses").
Bad Fit	• *high bias* • *high variance*	Unreliable and vague forecasts

### 4.5. Finding out how well the model performed with new data

Evaluations of models made use of unseen data that had yet to be considered throughout model construction. Seen data refers to information that has not been processed or utilised in any way. Additionally, unnoticed information has the potential to improve productivity and effectiveness by revealing areas of concern that need more attention. Actual information gathered from aviation crashes is made up of invisible data. In 2020, [42] was the source of the data. The amount of data collected was lower than that was utilised for the models. There are two theoretical buckets into which these undetected facts fall: normal and abnormal. The amount of unreported data is restricted to aircraft that occurred after 2003 and includes 1000 items of aberrant data and 1003 bits of regular data. Applying data that was not known before, the best model was 97 per cent accurate. Table 12 displays the disambiguation matrix outcomes. Whereas Table 13 shows the classification findings.

**Table 12:** An uncertainty matrix for the QDA model that was evaluated using hidden data.

*Parameter*		*Predicted Label*	
		*Normal*	*Abnormal*
*True Label*	*Normal*	961	42
	*Abnormal*	22	972

**Table 13:** Report on data classification for testing QDA prediction models with unseen data.

Parameter		Precision	False discovery rate	Recall	F1-score	Specificity	#Data
Normal	0	0.97	0.034	0.96	0.97	0.96	1003
Abnormal	1	0.96	0.025	0.97	0.97	0.97	1000
Accuracy		–	–	–	0.97	–	2003
Macro avg		0.97	0.03	0.97	0.97	0.96	2003
Weighted avg		0.97	0.03	0.97	0.97	0.96	2003

Several test criteria, including testing, training, cross-validating, ROC evaluation, and testing using unidentified information, show that the QDA system has attained excellent accuracy. Table 14 displays the accuracy data; the model is a solid fit, with a combined accuracy during training and testing of 0.93. With a cross-validation examination, the precision was found to be 0.94. The ROC, however, yielded values of 0.97 and 0.96, accordingly, when looking at the AUC findings for aberrant and healthy diagnosis. In other words, it proves that the ROC-based model is a "beneficial fit."

**Table 14:** Justification of the model using ROC and accuracy metrics.

Parameter	Training	Testing	K-Fold cross-validation	Unseen data	AUC Normal	AUC Abnormal	Remark
*Accuracy*	0.91	0.91	0.91	0.91	nagtive	nagtive	*Good Fit*
ROC	nagtive	nagtive	nagtive	nagtive	0.91	0.91	*Good Fit*

### 4.6. Independent expert confirmation

Table 15 shows that the top abnormality prediction model incorrectly predicted 25 out of 100 flight data points, the QDA classification model, which was tested with fresh data. After that, the professional pilots got their hands on the erroneous data, and they confirmed that all 25 erroneous data tags pointed to abnormal flying data, including height drop. Future pilots should keep climate and variations in direction and speed as potential causes of flying anomalies in mind. All three of these factors—velocity, guidance, and altitude—must be identical to the reference. For additional research, it is recommended to get experimental data.

**Table 15:** Comparison of results with previous approaches.

Study	Methodology	Accuracy (%)	Precision (%)	AUC	Key Features
[43]	Quadratic Discriminant Analysis (QDA)	**93**	**93**	**0.97**	High accuracy and precision; computationally efficient; real-time ADS-B data integration.
[44]	Isolation Forest (iForest)	89	85	0.92	Focused on energy anomaly detection; limited robustness to noise.
[45]	Digitization Programs + ADS-B	86	82	0.89	Emphasis on pilot safety; limited machine learning implementation.
[46]	Statistical Analysis of ADS-B Data	78	76	0.85	Statistical methods; no real-time application or ML integration.
[47]	Clustering-Based Anomaly Detection	81	80	0.88	Applied clustering for helicopter data; limited generalizability to fixed-wing aircraft.
[48]	Classification Using AWS Platform	84	83	0.87	Focused on differentiating flight operations; less anomaly detection emphasis

The proposed model demonstrates superior performance compared to previous approaches across key metrics such as accuracy, precision, and AUC. With an accuracy of 93% and an AUC of 0.97, the QDA-based model outperforms Isolation Forest and clustering-based approaches [49], highlighting its robustness and precision in anomaly detection. Unlike the statistical approaches used in studies such as [50], which lack predictive capability, the proposed model effectively integrates machine learning to detect anomalies proactively as shown in Table 15. Additionally, the proposed methodology’s reliance on real-time ADS-B data ensures practical applicability in commercial aviation, filling the gap left by approaches like [51], which focus on digitization programs without machine learning implementation. Moreover, while [52] achieved moderate success using clustering methods, the proposed model’s integration of QDA and expert-validated labeling techniques makes it better suited for general anomaly detection, particularly for fixed-wing aircraft. These comparisons demonstrate that the proposed approach not only advances the state-of-the-art in anomaly detection but also sets a new benchmark for integrating machine learning and real-time ADS-B data into aviation safety systems.

## 5. Theoretical and managerial implications

Both theoretical and practical settings may benefit from the flight anomaly forecasting framework that was created in this work. It consists of three parts. The flying abnormality-prediction software was built using AI, machine learning, and statistical methods. The research will advance in developing precise and practical algorithms for anticipating potential flight irregularities. Furthermore, the advancement of this model may enhance the understanding of the variables that lead to flight irregularities, including meteorological circumstances, human fallibility, and motor impairment. Furthermore, the process of developing and implementing models for prediction may serve to authenticate hypotheses about safety in aviation and enhance our comprehension of how deviations in flight might be avoided. The effects on management begin with the enhancement of safety. The use of the proposed flight abnormality-prediction system may assist carriers and aviation regulators in enhancing flight safety via the detection and prevention of prospective unusual occurrences. The implemented approach may also aid airlines in mitigating the expenses linked to flight irregularities, such as delays in flights, cancellations of flights, aircraft harm, and plane crashes (losses). Furthermore, the advanced prediction system may aid airlines in optimising flight operations and enhancing their effectiveness by accurately forecasting and preempting flight irregularities. Furthermore, enhancing the client experience will be achieved by offering greater accuracy on potential flight irregularities, as well as expedited and more efficient resolutions for consumers. Therefore, the advancement of flight anomaly prediction models is an expanding field of research that offers substantial advantages for the scientific and administrative elements of aircraft security and efficiency.

## 6. Conclusion

There were four main steps to the research methodology: problem definition, data curation, preprocessing of data, and data labelling. Then, a model for prediction was built and evaluated. During the launch and climb stages, the anomaly-detection system extracted data that was particular to commercial aeroplanes using the ADS-B data. For business trips using jet-engine aircraft, information has to be classified as the first category (Tier 1) due to its extraordinary quality. When it came to data labelling, the process followed the rules set down by the ICAO for jet-powered flights for business. Expert pilots who fly commercial aeroplanes checked the labels to make sure they were accurate. There were 167,844 flights in the dataset; 84,074 were considered regular, and 83,770 were deemed aberrant. Applying the imbalance ratio calculation to the dataset’s data showed that its attributes were balanced. The results showed that out of 25 models for prediction, the QDA model had the best accuracy at 0.93, indicating a very high degree of ability to predict. With an area under the curve (AUC) of 0.97 for aberrant identification and 0.96 for regular identification, the model was clearly a "good fit." This research focused on a single objective variable—height—and utilised machine learning approaches to predict unusual aircraft behaviour all through the takeoff and ascension stages. The forecasting model needs to make improvements to the three primary parameters in ADS-B data: direction, velocity, and height.

## List of abbreviations

ADS-B: Automatic Dependent Surveillance-Broadcast
AI: Artificial Intelligence
ML: Machine Learning
FDR: Flight Data Recorder
CVR: Cockpit Voice Recorder
ICAO: International Civil Aviation Organization
AUC: Area Under the Curve
QDA: Quadratic Discriminant Analysis
FOQA: Flight Operations Quality Assurance
AWS: Amazon Web Services
SME: Subject-Matter Experts
FAA: Federal Aviation Administration
ATPL: Airline Transport Pilot License
ROC: Receiver Operating Characteristic
F1-score: A measure of a test’s accuracy considering precision and recall
DFDR: Digital Flight Data Recorder
SSR: Secondary Surveillance Radar
TPs: True Positives
TNs: True Negatives
FPs: False Positives
iForest: Isolation Forest Algorithm
ADS-B Out: ADS-B Transmitter
